# Cultivation of College Basketball Referee Ability Using Infrared Thermal Imaging Target Recognition and Tracking System

**DOI:** 10.1155/2022/8936973

**Published:** 2022-07-15

**Authors:** Dezhu Li

**Affiliations:** Department of Physical Education, Yuncheng University, Yuncheng 044000, China

## Abstract

With the development of economy and culture and the improvement of infrastructure, basketball is becoming more and more popular. At the same time, whether in school or society, basketball events are increasing, and the demand for basketball referees is also rising. As the base and cradle of training basketball referees, colleges and universities are important places for incubating basketball referees. However, the basketball referee ability cultivated in colleges and universities is still lacking, which cannot meet the increasingly standardized basketball events and basketball training. Infrared thermal imaging has the characteristics of passive imaging, high recognition accuracy, and strong anti-interference. It is especially suitable for tracking and testing basketball players, and this is expected to further improve the comprehensive ability of basketball referees. Based on this, a target recognition and tracking system based on infrared thermal imaging is proposed in this study. Its purpose is to use it to carry out comprehensive ability training for college basketball referees. Experiments show that target recognition and tracking based on infrared thermal imaging can improve the comprehensive ability of basketball referees by 40.32%, and the awareness of basketball referees to fouls has also reached 88.6%. This fully shows that the target recognition and tracking system based on infrared thermal imaging can effectively improve the comprehensive ability of basketball referees and make basketball more regular and standardized.

## 1. Introduction

With the surge of national sports, basketball has gradually entered thousands of households. Basketball referees are the core of basketball, but with the increasing number of competitions, the speed of training basketball referees in colleges and universities cannot keep up with the changing demand. Moreover, basketball referees trained based on theory cannot adapt to the standardized and standardized basketball game. Infrared thermal imaging can realize target recognition and tracking. Based on this, a target recognition and tracking system based on infrared thermal imaging technology is proposed in this study. It aims to continuously promote the comprehensive ability of basketball referees. On the one hand, enhancing the comprehensive ability of basketball referees can promote the continuous normalization of the game and ensure the smooth progress of various sports. On the other hand, target recognition and tracking based on infrared thermal imaging can provide new ideas for the development of other fields. It also continuously optimizes the original structure and system and finally speeds up the upgrading rhythm of the industry.

After a series of experimental analysis, we can know that the target recognition accuracy based on infrared thermal imaging technology is relatively high, up to 91.23%. The accuracy of target recognition based on the general algorithm is only 90.22%. Moreover, with the increase of the number of people in the image, the recognition accuracy of the two methods is declining, and the recognition accuracy of the general method is up to 3%. At the same time, target recognition and tracking based on infrared thermal imaging technology play a certain role in improving the comprehensive ability of basketball referees. Among them, this technology can first improve the computer level and English level of basketball referees and their professional ability, with a maximum increase of 29.1%. Second, the technology can also enhance the basketball referee's understanding of various rules, in which the referee's mastery of the rules has increased by nearly 43.9%. Finally, target recognition and tracking based on infrared thermal imaging technology can also enhance the psychological quality of basketball referees and prevent them from stage fright, in which the comprehensive psychological quality has been improved by 10%. This fully demonstrates that target recognition and tracking based on infrared thermal imaging can effectively promote the training of basketball referee ability in colleges and universities and finally establish a professional team of referees.

## 2. Related Work

With the popularization of basketball, more and more colleges and universities begin to train their own basketball referees to form their own basketball teams. At the same time, many experts and scholars have focused their attention on this.

Candra et al. aimed to determine the impact of a basketball referee's physical condition on his or her refereeing ability. In the course of the study, he used a quantitative method and randomly selected 12 basketball referees to assess their physical condition. The results show that the average score of basketball referees' physical condition is 8.3, belonging to the middle category [1]. Karaam and Pulur aimed to examine the relationship between referee self-efficacy and general self-efficacy of basketball referees in terms of gender, education, age, and referee experience. During this process, he used the Referee Self-Efficiency Scale (REFS) and General Self-Efficiency Scale (GSE) as data collection tools and analyzed the data using the SPSS 21 and AMS programs [2]. Paula et al. pointed out that a basketball referee is the authority responsible for ensuring that rules and regulations are followed and decisions are made, so the physical and psychological qualities of the referee are essential for good performance on the field. To fully understand the health and psychological problems faced by basketball referees, he conducted a prospective cohort study. He also used standardized forms to evaluate the overall quality of basketball referees [3]. Faruk and Ilkay aimed to study the physical condition, physical preparation, and specific psychological preparation of basketball referees when they are present. Based on this, he designed a system to detect and evaluate the overall quality of basketball referees and made a comparative analysis of basketball referees from the gender level [4].

The above experts and scholars have analyzed the physical and psychological qualities of basketball referees from different levels, but they have not put forward specific methods to improve basketball refereeing ability. Infrared thermal imaging can be used to track and detect basketball players and provide technical support for referees to improve their self-ability. Therefore, the following articles will refer to the literature related to infrared thermal imaging.

Oliveira et al. proposed a tip thermal infrared enthalpy (in-tip TIE) method for fast enthalpy analysis. In this approach, he suggested that temperature monitoring by an infrared camera can be combined with the response within the suction head of a multichannel liquid dispenser. Among them, the filter paper can be used inside the suction head to retain the reagent as a solution or solid for neutralization, redox, or precipitation reactions [5]. Sousa et al. proposed that infrared thermal (IRT) imaging is a medical imaging mode to study skin temperature in real time, which can provide useful diagnosis and monitoring information of directly or indirectly related diseases. At the same time, he pointed out that one of the most accessible body parts for research using this imaging method is the hand, which can reflect all the information about the condition of the upper limbs. In order to understand the successful application of IRT in the medical field and open up a vision for future application according to the results obtained, he took the lead in creating the application of IRT in the hand [6]. Zhang and Guo pointed out that the key laboratories of chemistry on campus, especially the key laboratories of pharmacy, are high‐risk areas for safety accidents. In order to effectively reduce or even eliminate safety risks and reduce the risk of safety accidents, he proposed to design a sentinel robot equipped with infrared thermal imaging module. The robot can take appropriate emergency measures to detect dangerous situations, including alarm and firefighting, so as to minimize accidents and reduce economic losses [7]. Jung et al. pointed out that infrared thermography has been widely used to show the correlation between body thermal characteristics and muscle activation. To this end, he aimed to study a method of using thermal imaging to visualize and distinguish target muscles during resistance training. During the experiment, he segmented and converted the obtained thermal images into thermal maps and then generated differential thermal maps from paired thermal maps [8].

The above scholars have carried out detailed research on thermal imaging technology and have innovated it in different fields. However, in this process, they have not applied this technology to the field of sports, so its research has some limitations.

## 3. Infrared Thermal Imaging Target Recognition and Tracking and Cultivation of College Basketball Referee Ability

### 3.1. Infrared Thermal Imaging

In the normal atmosphere, the wavelength of visible light of human eyes is between 0.4 and 0.75 *μ*m and the electromagnetic wave with a wavelength between 0.75 and 10000 *μ*m is called infrared wave, which cannot be directly observed by human eyes [9]. Among them, the infrared wave with a wavelength between 0.78 and 2.0 *μ*m is called near infrared. The band of infrared thermal imaging discussed in this study is mainly between 3 and 5 *μ*m. The spectra of visible and invisible light are shown in Figure 1.

Any object whose temperature is higher than absolute zero will emit infrared energy according to its temperature. The infrared energy emitted by the object is called thermal characteristic. Generally speaking, the hotter an object is, the more radiation it emits. Infrared thermal imaging is essentially a thermal sensor, which can detect and capture small temperature changes [10]. It collects infrared radiation from objects in the scene, creates pixels, and forms an image according to the information about the temperature difference. Because objects rarely have the same temperature as the surrounding objects, the thermal imager can detect the difference and produce a sharp contrast in thermal imaging, which is the basic principle of infrared thermal imaging. An infrared thermal imager was first used in the military, as it can detect objects in a completely dark environment. Even in the case of smoke and dust, it does not need a visible light source. Therefore, it can be used 24 hours a day. The thermal imager passively detects the infrared radiation emitted by objects, which is more hidden than other active imaging systems with light sources. Due to its good concealment and strong anti-interference ability, strong target recognition ability, and adaptability, the infrared thermal imager is often used in military intelligence, surveillance, and guidance, and is widely used in weapons and equipment [11].

In the postspecial period, as the most important epidemic prevention temperature measuring equipment, the infrared thermal imager has more and more prominent advantages in safety [12]. Based on this, the trend of using infrared thermal image temperature measurement equipment has rapidly swept all industries in recent years. The infrared thermal imager has become a strong application in more and more fields because of its advantages of fast accurate identification, wide environmental adaptability, and strong infrared penetration. The main application fields of infrared thermal imaging are shown in Figure 2.

With the progress and development of science and technology, infrared thermal imaging technology is also upgrading. At present, the wafer is cut into a single chip for packaging. With the gradual maturity of wafer-level packaging and 3D packaging, the packaging process of overall packaging before cutting can be realized in the future. The new packaging process can greatly improve the scale effect and production efficiency and effectively reduce the packaging cost. In recent years, some manufacturers have taken the lead in developing ASIC chip integration rather than PCB circuit board level component integration, which greatly reduces the size and mass production cost of imaging modules [13]. In the future, with the large-scale production of products integrated with ASIC, the scale effect will be more significant, and more manufacturers in the industry will adopt this technology. With the rapid development of emerging economies, the infrared thermal imager has become an important consumer market in the civil field. The infrared thermal imager can be applied to the fields of infrastructure construction, urban management, industrial production, traffic control, and resource exploration in emerging economies. In the macromarket, with the adjustment of economic structure and the continuous growth of economy, the infrared thermal imager will play a greater role in the process of industrial modernization, such as modern industrial production fields, including industrial testing, manufacturing management, and electrical automation, as well as urban monitoring, inspection and quarantine, and fire safety in urban construction in the future [14]. The classification of infrared thermal imaging is listed in Table 1.

### 3.2. Target Recognition and Tracking

In the early field of computer vision, target tracking is usually described as following interest points in a short space. Because the early time tracker is simple, fast, and robust, the early tracking usually adopts the time tracking strategy. However, without strong low-level clues such as corner and peak intensity, target tracking is easy to fail [15]. Therefore, with the birth of high-performance target detection mode, a powerful alternative method appears, that is, the target detection tracking method. In practice, the target detection and tracking model can rely on the given accurate recognition rate to determine the target objects, and then they are connected according to time series from another stage.

Detection-based tracking generally uses the target detector based on deep learning, which is the mainstream target tracking paradigm at present. However, the target tracker with the best performance is not without disadvantages [16]. Many trackers need to rely on low-speed and complex correlation strategies to connect the detection frames in series according to time. Infrared thermal imaging tracking technology is a passive target detection and tracking technology, which is used for target detection, extraction, and tracking of infrared video signal. Contrast feature recognition is a common target extraction method. The algorithm cannot remember and recognize the morphological features of the target, and the extraction effect and tracking stability are poor in complex background. The template matching algorithm takes the target feature data as the template and looks for matching points in the search area, that is, taking the target shape feature as the criterion to realize target retrieval and tracking. Even in complex background, the tracking sensitivity and stability are very high, which is very suitable for target tracking in complex background.

Infrared thermal imaging can avoid the influence of illumination and other factors and improve the accuracy of object recognition. However, the image obtained by the infrared thermal imager has a high gray level, so it often has a lot of noise. Therefore, in order to effectively carry out target recognition, we first need to process the image. The smoothing filter is usually used to denoise the image, and its mathematical expression is as follows:

(1) $$\begin{array}{c} g\left(x,y\right)=\frac{1}{N}\sum_{i,j\in S}f\left(i,j\right). \end{array}$$

In the above formula, *g*(*x*, *y*) represents any point in the image area, and *N* represents the midpoint of the area. From the above expression, we can see that the smoothing filter will blur the image in the process of noise reduction and then lose a lot of image information. A low-pass filter is an upgrade of smoothing filter, which can effectively retain the effective information in the image. Its mathematical description is as follows:

(2) $$\begin{array}{c} G\left(i,j\right)=J\left(i,j\right)•F\left(i,j\right),\\ J\left(i,j\right)={\left[i^{2}+j^{2}\right]}^{1/2}. \end{array}$$

*J*(*i*, *j*) is the core function of the low-pass filter, and the result can be obtained only after two Fourier transforms. The transformation process of the core function is shown in Figure 3.

A median filter can deal with some nonlinear noise problems, which can effectively suppress salt and pepper noise. In the process of image denoising, the median filter can not only remove the noise but also ensure the integrity of image information and restore the image to its original state. Compared with a low-pass filter, the biggest advantage of median filter is that it can deal with the isolated noise in the image and make the image more realistic. Its mathematical expression is as follows:

(3) $$\begin{array}{c} z_{ij}=\text{Med}\left\{x_{ij}\right\}\\ =\text{Med}\left\{x_{\left(i+r\right)\left(j+r\right)},\left(r,s\right)\in A,\left(i,j\right)\in I^{2}\right\}. \end{array}$$

In the above formula, *A* refers to the neighborhood of point *x*_*ij*_ and *I* refers to the independent point set. In the image, the selected points are different, and their fields will change accordingly, so how to partition is very important.

Assuming that there are *n* data points in the image, these data points constitute a certain functional relationship. In order to express the relationship between points, we define a kernel density function, which is expressed as follows:

(4) $$\begin{array}{c} f\left(x\right)=\frac{1}{n}\sum_{i=1}^{n}K_{H}\left(x-x_{i}\right),\\ K_{H}={\left|H\right|}^{\left(1/2\right)}K\left(H^{-\left(1/2\right)}x\right). \end{array}$$

In the above formula, *H* represents the bandwidth and *K* represents the kernel function, which is mathematically described as the frequency of isolated points in the unit interval. In particular, kernel functions are generally asymmetric and converge in the domain of definition.

The emergence of bandwidth makes the image processing process more complex, so we need to simplify this method and reduce unnecessary workload. The improved nuclear density can be expressed as follows:

(5) $$\begin{array}{c} f_{k}=\frac{c_{k}}{nh}\sum_{i=1}^{n}\left({\left|\left|\frac{x-x_{i}}{h}\right|\right|}^{2}\right),\\ h=K\left(x\right)\\ =k\left({\left|\left|x\right|\right|}^{2}\right),\\ n=\int_{0}^{\infty }k\left(r\right)\text{d}r<\infty . \end{array}$$

In the above formula, *k* is nonnegative and monotonic in the domain. On this basis, the image processing is basically simplified. Next, we need to model and track the target. In the initial image, we will weigh the target to be detected according to the kernel function, in which the weight of the pixel near the center point is large and the weight of the pixel far away is small. The objective model function is expressed as follows:

(6) $$\begin{array}{c} q=C\sum_{i=1}^{n}k\left({\left|\left|\frac{x_{i}-x_{0}}{h}\right|\right|}^{2}\right)\delta \left[b\left(x_{i}\right)-u\right], \end{array}$$

where *x*_0_ is the midpoint coordinate of the image, *C* is a constant, and *b*(*x*) represents the attribute of the target area. After modeling the target model, we also need to model the candidate regions to ensure the real-time tracking of the target.

The candidate target model can be expressed as follows:

(7) $$\begin{array}{c} p=C\sum_{i=1}^{n}k\left({\left|\left|\frac{x_{i}-y}{h}\right|\right|}^{2}\right),\\ y=\sum_{u=1}^{m}\left[p\left(x\right)-u\right]. \end{array}$$

After having the target model and candidate model, it is much easier to realize the target tracking. In the process of target tracking, the similarity between the two models describes the predicted position of the target. The similarity between models is calculated as follows:

(8) $$\begin{array}{c} \theta =\rho \left[p\left(y\right),q\right]\\ =\sum_{u=1}^{m}\sqrt{p_{u}\left(y\right)q}, \end{array}$$

where *θ* represents the similarity, and its value is between 0 and 1. Among them, the larger the coefficient, the greater the similarity between the actual target and the predicted target, and the smaller the coefficient, the smaller the similarity between the targets. Taylor expansion calculation is carried out for the above formula at *y*_0_ point, and the results are as follows:

(9) $$\begin{array}{c} \rho \left[p\left(y\right),q\right]\approx \frac{1}{2}\sum_{u=1}^{m}\sqrt{p_{u}\left(y_{0}\right)q}+\frac{1}{2}\sum_{u=1}^{m}p_{y}\left(y\right)\sqrt{\frac{q}{p\left(y_{0}\right)}}. \end{array}$$

From the above formula, we can see that the similarity of the second term can affect the similarity of the whole function, so we use the mean shift method to enlarge it to get

(10) $$\begin{array}{c} y=\frac{\sum_{i=1}^{n}x_{i}w_{i}g\left({\left|\left|y-x_{i}/h\right|\right|}^{2}\right)}{\sum w_{i}g\left({\left|\left|y-x_{i}/h\right|\right|}^{2}\right)},\\ w_{i}=\sum_{u=1}^{m}\gamma \left[b\left(x_{i}\right)-u\right]\sqrt{\frac{q_{u}}{p_{u}\left(y\right)}}. \end{array}$$

Among them, the above formula is a new target point obtained by the mean shift method, *y*_0_ is the target center point, and *w*_*i*_ is the target weight. When ||*y*_1_ − *y*_2_|| < *ε* occurs, target matching ends and the final result is generated. A basic target recognition and tracking system based on infrared thermal imaging has been established.

### 3.3. Training of Basketball Judging Ability in Colleges and Universities

Basketball is deeply loved by the people, with a strong mass base, so basketball also has more appreciation. When people participate in competition, they can often improve their own competitive strength, so they have a strong interest [17]. Basketball referees, as “referees” on the court, are also the specific executors of the rules of the game, and they are an indivisible key part of basketball. In order to better develop basketball activities, we must constantly train basketball referees at all levels and technical levels. A reasonable, fair, and correct referee system can ensure the smooth development of basketball, and the execution level of basketball referees directly affects the quality and results of basketball matches [18].

Basketball referees have the right to adjudicate violations of the rules, whether within or outside the boundaries, including the record table, team seats, and areas close to the bottom line. The basketball referee should whistle when there is a violation of the rules, when the game is over, or when the basketball referee considers it necessary to interrupt the game. Basketball referees should not whistle after a successful shot, a free throw, or a ball has survived. Basketball referees should pay attention to and consider the following basic principles when determining physical contact or violations:

1. The spirit and intent of the rules and the need to adhere to the integrity of the game.
2. Using the consistency of this concept, the basketball referee should not attempt to penalize accidental physical contact by unnecessarily interrupting the fluidity of the match. In addition, such contact will not benefit responsible participants or be detrimental to other participants.
3. Using consistency of common sense in each competition.

Basketball has a broad mass base. It is a kind of ball that both boys and girls can play. It is deeply welcomed by the majority of students. In a basketball match, the basketball referee is responsible for the battle between the two sides. In the course of the match, the two referees work together to achieve the best combination of free-throw techniques on the field [19]. However, the basketball referee's judgment should also have a standard. The referee's behavior should conform to the basketball rules and the basketball referee law to ensure that both teams play smoothly under fair and fair conditions. However, in the actual adjudication process, due to various reasons, basketball referees often cannot effectively record and discover violations. At the same time, due to the referees' own reasons and group attributes, their referee process often lacks some supervision and restriction, which also brings challenges to basketball referees. The diagram of the auxiliary tools used by the basketball referee on the spot is shown in Figure 4.

In basketball, the absence of players and referees cannot be a wonderful basketball feast, so training professional basketball players and referees is the premise of developing basketball matches [20]. However, for the current stage of sports students, their ability to refer to basketball is still quite weak. So, their basketball execution is poor or none, let alone their experience in refereeing on the spot. To cultivate the basketball referee ability of college physical education students, we must master the rules and methods of basketball referee. In order to solve this problem, colleges and universities teach basketball rules and basketball referees to all students of physical education specialty. This is to find potential in schools. They focus on training the actual students of basketball referees, so that they can learn basketball referee skills in depth.

In the specific implementation process, universities should first select suitable candidates and focus on training their comprehensive ability. After all the judges have been selected, what the school needs to do next is to train them with strict theoretical knowledge, because a qualified and excellent basketball referee must master all aspects of basketball referee theoretical knowledge. Therefore, in the teaching of basketball theory, colleges and universities will arrange teachers to give detailed lectures on the theoretical knowledge of basketball referee rules and basketball referee methods and ensure that students have all the knowledge, and teachers will also open classroom tests at random. The most important thing in basketball judging is the cultivation of gestures. During the training of gestures and whistles, teachers should explain and demonstrate each gesture and whistle in detail and explain the function and significance of each gesture and whistle. At the same time, with the development of science and technology, the basketball referees should keep up with the times and master the latest science, technology, and methods. For this reason, we studied the basketball coach's computer skills, and the results are shown in Figure 5.

Figure 5 shows that male basketball referees are generally better at computer than female basketball referees. Of these, 25% of the male referees can fully master the computer operation, but only 12% of the female referees can fully master the operation. Moreover, 15% of the referees said they were unfamiliar with computer operations.

On the basis of theoretical knowledge, students have preliminarily qualified to be a basketball referee, but practice is the only standard to test the truth, so the next school should also examine it in practice. In this process, students can practice not only in the classroom but also after class. Practice can run on the basketball court to simulate the situation of the court or practice many times against the mirror to achieve beautiful and generous gestures. The referee's gestures are essential from the beginning to the end of a basketball match. This is the most intuitive judgment because it clearly reflects the players' violations on the field. The referee's gestures are often used to communicate information between two basketball referees, between a basketball referee and a basketball coach, between basketball players, and between a basketball referee and a recorder. Therefore, they must use gestures correctly in basketball matches. Any judgment should be based on the basketball referee's gesture, so as to achieve the combination of gesture and language. But at the same time, the referee must ensure that the verdict gestures are clear, decisive, graceful, and generous. However, different factors will affect their referee level, among which the factors that affect the basketball referee's judgment are listed in Table 2.

Table 2 lists that the mastery of rules will directly affect the judgment of referees, of which 32% of referees said that the situation of rules is a major factor affecting their judgment. At the same time, the referee's own quality and English level will also directly affect the referee's judgment, of which the highest degree of influence can reach 44%.

## 4. Effect of Infrared Thermal Imaging in Cultivation of Basketball Referee Ability

In order to explore the utility of infrared thermal imaging technology in the actual training process, we conducted a simple experiment on the class carrying out basketball training. Because infrared thermal imaging is passive imaging, no one intervened to destroy the experiment in the whole process of the experiment. At the same time, in order to improve the imaging quality of infrared thermal imaging, we first use the filter to simply process the image and then recognize and track the target on the basis of the built model. Among them, the target recognition using the infrared thermal imaging technology proposed in this study is listed in Table 3, and the target recognition using the general algorithm is listed in Table 4.

Experiments show that this study also carries out image recognition and tracking on 50 images, and different methods have different effects. Among them, the target recognition accuracy based on infrared thermal imaging technology is relatively high, up to 91.23%, while the target recognition accuracy based on the general algorithm is only 90.22%. Moreover, with the increase of the number of people in the image, the recognition accuracy of the two methods is declining, and the recognition accuracy of the general method is up to 3%.

The above experiments clearly show that the target recognition based on infrared thermal imaging technology has significant advantages, but it cannot explain its effectiveness in the actual cultivation of basketball referee ability. Based on this, the article will continue to explore its role in practice, which aims to further prove the effectiveness of this method in the cultivation of basketball referee ability.

The skills of gesture, whistle blowing, and the application of rules are the basic skills that basketball referees should have. In order to explore the effect of infrared thermal imaging technology, we studied it from the basic skills. Among them, Figure 6 shows the basketball coach's mastery of basic skills.

Figure 6 shows that, compared with the original situation, the target recognition and tracking based on infrared thermal imaging technology can greatly help the referee to judge and remember. Among them, the basic gesture mastery of basketball referees increased from 60 to 112, an overall increase of 80%. Moreover, for illegal dribbling, alternating possession, and other fouls, the referee can more intuitively observe the specific actions and master the key points. Among them, its mastery increased from 60 to 90, a year-on-year increase of 33%.

By judging the basic skills of basketball referees, we can find that target recognition and tracking based on infrared thermal imaging technology can play a certain effect in the actual training process. But basic skills represent the basic skills of referees. General basketball referees can improve slowly without relying on special skills, so their representativeness is not strong. It is the most important ability of basketball referees to judge and deal with fouls in time. It can represent the overall quality of basketball referees authoritatively. Therefore, we studied the cognition of basketball referees on foul behavior before and after the experiment, and the results are shown in Figure 7.

Figure 7 shows that there are obvious differences in basketball referees' cognition of foul behavior before and after the experiment. Among them, basketball referees' cognition of basic foul behaviors such as walking with the ball has been increased to 80%, and their cognition of free ball has also been increased to 90%. This fully shows that target recognition and tracking based on infrared thermal imaging technology can effectively improve the basketball referee's cognition of foul behavior and improve the basketball referee's ability.

From the above experiments, we can know that target recognition and tracking based on infrared thermal imaging technology can effectively improve the ability of basketball referees. In order to explore its comprehensive impact on basketball referee ability, we compared the comprehensive ability of basketball referee before and after the experiment, and the results are shown in Figure 8.

Figure 8 shows that target recognition and tracking based on infrared thermal imaging technology play a certain role in improving the comprehensive ability of basketball referees. Among them, this technology can first improve the computer level and English level of basketball referees and their professional ability, with a maximum increase of 29.1%. Second, the technology can also enhance the basketball referee's understanding of various rules, in which the referee's mastery of the rules has increased by nearly 43.9%. Finally, target recognition and tracking based on infrared thermal imaging technology can also enhance the psychological quality of basketball referees and prevent them from stage fright, in which the comprehensive psychological quality has been improved by 10%.

## 5. Conclusion

Extracurricular learning can help students cultivate their interest and vision in basketball refereeing, and activity practice can help college students turn their refereeing knowledge and skills into practical experience. Taking the basketball referee's ability as the starting point, this study aims to promote colleges and universities to strengthen the training of basketball referees. On this basis, starting with infrared thermal imaging technology, this study first analyzes the characteristics and development of infrared thermal imaging and then further proposes an image recognition and tracking system based on infrared thermal imaging technology. Then, the study further analyzes the effectiveness of recognition and tracking based on infrared thermal imaging technology on the cultivation of basketball referee ability. Finally, the relevant experiments are designed, analyzed, and summarized in detail. It fully shows that target recognition and tracking based on infrared thermal imaging technology can play a certain role in improving the comprehensive ability of basketball referees. However, due to time reasons, the article did not make a specific analysis of other abilities of basketball referees. In the future, the article will comprehensively analyze the various abilities of basketball referees and constantly promote their all-round development.

## Figures and Tables

**Figure 1:** Visible and invisible light spectra.

**Figure 2:** Application field of infrared thermal imaging.

**Figure 3:** Transformation process of core function.

**Figure 4:** Diagram of basketball referee's on-the-spot assistant tool.

**Figure 5:** Computer mastery of basketball coach.

**Figure 6:** Basketball coach's mastery of basic skills.

**Figure 7:** Basketball referee's cognition of foul behavior.

**Figure 8:** Improvement of comprehensive ability of basketball referees.

**Table 1:** Classification of infrared thermal imaging.

	Not cooled infrared thermal imaging	Cooled infrared thermal imaging

Principle	Thermal effect	Photoelectric effect
Advantage	Small volume	High sensitivity
Shortcoming	Low sensitivity	Low temperature environment
Application scenarios	Military and civilian	Aerospace

**Table 2:** Factors influencing basketball referees' judgment.

Factor	Degree	Percentage (%)

Rule	Big	32
Off-site factors	Generally	20
Personal reasons	Larger	44
English language proficiency	Larger	38
Computer skill	Small	2
Other	Small	5

**Table 3:** Target recognition of infrared thermal imaging in basketball training.

Test sequence	Number of image	Number of people	Detection rate	Operation hours

1	50	15	91.23	1.365
2	50	19	91.11	1.651
3	50	25	93.25	1.789

**Table 4:** Target recognition of general algorithms in basketball training.

Test sequence	Number of image	Number of people	Detection rate	Operation hours

1	50	14	90.22	1.365
2	50	20	88.27	1.651
3	50	25	87.36	1.789

## Data Availability

The data used to support the findings of the study can be obtained from the author upon request.
